# Design of Knowledge Graph Retrieval System for Legal and Regulatory Framework of Multilevel Latent Semantic Indexing

**DOI:** 10.1155/2022/6781043

**Published:** 2022-07-19

**Authors:** Guicun Zhu, Meihui Hao, Changlong Zheng, Linlin Wang

**Affiliations:** ^1^Department of Economic Management, Dongchang College of Liaocheng University, Liaocheng 252000, Shandong, China; ^2^Dongchang Middle School of Liaocheng Economic and Technological Development Zone, Liaocheng 252000, Shandong, China; ^3^Liaocheng Yucai School, Liaocheng 252000, Shandong, China

## Abstract

Latent semantic analysis (LSA) is a natural language statistical model, which is considered as a method to acquire, generalize, and represent knowledge. Compared with other retrieval models based on concept dictionaries or concept networks, the retrieval model based on LSA has the advantages of strong computability and less human participation. LSA establishes a latent semantic space through truncated singular value decomposition. Words and documents in the latent semantic space are projected onto the dimension representing the latent concept, and then the semantic relationship between words can be extracted to present the semantic structure in natural language. This paper designs the system architecture of the public prosecutorial knowledge graph. Combining the graph data storage technology and the characteristics of the public domain ontology, a knowledge graph storage method is designed. By building a prototype system, the functions of knowledge management, knowledge query, and knowledge push are realized. A named entity recognition method based on bidirectional long-short-term memory (bi-LSTM) combined with conditional random field (CRF) is proposed. Bi-LSTM-CRF performs named entity recognition based on character-level features. CRF can use the transition matrix to further obtain the relationship between each position label, so that bi-LSTM-CRF not only retains the context information but also considers the influence between the current position and the previous position. The experimental results show that the LSTM-entity-context method proposed in this paper improves the representation ability of text semantics compared with other algorithms. However, this method only introduces relevant entity information to supplement the semantic representation of the text. The order in the case is often ignored, especially when it comes to the time series of the case characteristics, and the “order problem” may eventually affect the final prediction result. The knowledge graph of legal documents of theft cases based on ontology can be updated and maintained in real time. The knowledge graph can conceptualize, share, and perpetuate knowledge related to procuratorial organs and can also reasonably utilize and mine many useful experiences and knowledge to assist in decision-making.

## 1. Introduction

With the rapid development of Chinese society and the continuous improvement of the legal system, the number of cases heard by courts across the country has increased year by year, and judges accept more than 100 cases per year on average [1]. In addition, due to the advancement of the reform of the litigation system, case handlers are required to avoid differences in trials caused by personal factors while ensuring the efficiency of case-handling so as to ensure the fairness of the case [2]. Under the multiple constraints, the work pressure on case investigators is increasing day by day. How to scientifically and effectively improve the efficiency and fairness of judicial cases has become an urgent problem to be solved. “Smart Court” is a concept proposed by the leading group of the Supreme People's Court informatization construction [3]. It mainly uses modern artificial intelligence technology, adheres to the correct judicial concept, combines judicial laws with various reforms, and builds the judicial system with a high degree of informatization. In accordance with the basic work path of informatization instructed by superior leaders, the court has made excellent progress in the network, sunshine, and intelligence of smart courts [4].

As a relatively cutting-edge technology in natural language processing tasks, knowledge graphs have great potential in the construction of court informatization [5]. It is a technical method that uses graph models to describe knowledge and build relationships between things. Knowledge graphs are divided into two categories. General knowledge graphs are the most common and most used type of knowledge graph because of their wide knowledge coverage and many fields [6]. Domain knowledge graphs are mainly aimed at specific fields, emphasizing the depth of knowledge. In view of the complex and rigorous knowledge characteristics of the judicial field, it is a better choice to build a knowledge graph in the field of legal documents. At the same time, the maturity of machine learning and the maturity of graph databases have provided strong support for the construction of legal document knowledge graphs [7].

As far as the judiciary is concerned, there are various types of massive data, such as laws and regulations, judgment documents, and domain knowledge. Building a knowledge graph can satisfy data association, knowledge expansion, and application support [8]. The judicial knowledge graph is the basis for the intelligent application of legal supervision agencies; a properly structured judicial knowledge graph is the key to promoting judicial intelligence. Data is a resource that is independent of the others. Only when these resources are used effectively can data reflect its true value. The deep integration of big data technology and judicial knowledge can effectively promote the informatization transformation of procuratorial organs [9]. On the one hand, the research on the intelligent procuratorial case-handling assistance system based on the knowledge graph can integrate the knowledge graph technology into judicial case-handling so as to realize the informatization, systematization, and shared management of judicial knowledge, which is helpful for the concealment of judicial knowledge. The information is analyzed and mined to realize secondary utilization. On the other hand, the research on the intelligent procuratorial case-handling assistance system based on the knowledge graph also provides technical support means for optimizing case-handling and assisting decision-making [10].

This paper analyzes the Zipf law of singular value distribution in latent semantic space and its statistical significance. Then, based on the power approximation method and Ding's double probability model, the hidden statistical properties of word (document) vectors are deeply analyzed. Dimensions corresponding to large singular values represent more “commonality” and less “personality” of language elements, while dimensions corresponding to small singular values represent more “personality” and less “commonality” of language elements. This paper introduces the operation syntax and storage method based on the Neo4j graph database and designs a knowledge graph system based on the public domain of procuratorial affairs. It is based on the Spring Boot framework and explains the function and characteristics of each functional module in the system. The system interface and the knowledge graph are used to make the query results and result display structured and improve the search experience. The theories of CRF, RNN, LSTM, bi-LSTM, and bi-LSTM-CRF are introduced, and the structure of each model is analyzed. Experiments show that the model proposed in this paper has achieved a significant improvement in the task of crime prediction, which verifies the effectiveness of our proposed method. In this paper, the test results of the relevant application functions of the test system are given, and the verification and analysis are carried out.

## 2. Related Work

Relevant scholars elaborated on the application of legal knowledge graphs in the field of judicial artificial intelligence [11]. He took fact-based civil judgments as his research goal and came to the conclusion that artificial intelligence technology at its emerging stage has not yet reached the technical level that can replace judges. The researchers discussed the construction method of the “smart court” knowledge system and explained the importance of modern information technology and the difficulties in the construction of knowledge graphs [12].

Entity extraction can also be called entity recognition. Its main task is to extract specific entity information elements from text, which is the basis for building knowledge graphs. The research on entity extraction problems has a long history, and the existing methods can be generally divided into rule-based, statistics-based, and deep learning-based methods [13].

Rule-based methods usually rely on relevant experts, use professional knowledge to construct rules manually, and can provide reference features such as statistical information, punctuation marks, and keywords. The number of entity extraction rules usually obtained by such methods is very large, and then the rules are extracted. Matching with the characters in the text to achieve the effect of identifying the entity, it has the advantages of low algorithm complexity, simple method, and simple implementation [14].

The c-TAKES dictionary played an important role in entity recognition tasks in the early biomedical field by extracting information from electronic clinical medical record texts to construct an open-source natural language processing system. This entity extraction method has been experimentally proved that it has excellent performance on small datasets, but as the dataset continues to increase, the scope of the rules is getting smaller and smaller, and the rules need to be supplemented at a great artificial cost [15]. Moreover, the portability of this method is poor, and the application of the same set of rules in different fields varies greatly.

Related scholars use the maximum entropy model to use the short-term rating data set on Twitter (a social networking service platform) and propose a method to discover the contextual clustering of microtexts by using three properties of contextual associations between microtexts [16]. Relevant scholars have proposed a CRF-based entity recognition method, which considers the fine-grainedness of candidate entities by using two levels of word-based and character-based segmented text and extracts according to the feature templates trained in the training phase [17].

Based on the cyclic neural network combined with the conditional random field model, relevant scholars have focused on the splicing of word vectors and character vectors, adding an additional attention mechanism so that the model can dynamically use the vector information to change the parameter weights and further improve the performance of entity recognition [18]. For entity extraction of legal documents, related scholars proposed a novel method based on a pretrained model, which completed the sequence labeling task by learning large-scale real data from Brazilian legal documents [19]. A scalable sequence tagging model named sequence tagging model (STM) has been developed, and extensive experiments verify the effectiveness of STM for entity extraction tasks [20].

Relevant scholars used kernel functions in entity relation extraction tasks and introduced their calculation method [21]. Combined with SVM classifier and perceptron, two hundred news corpus were used as data, and good results were obtained. The disadvantage of the method based on feature vector is that the generalization is poor, the extraction effect of the same model for different fields is very different, and the selection of features also greatly affects the performance of the model. The disadvantage of the kernel function is that the computational complexity is high, the model training time is long, and the performance of the model also depends on the selection of features [22].

Taking the scope of knowledge covered as an indicator, knowledge graphs are divided into general-purpose and vertical domain knowledge graphs [23]. The general knowledge graph contains a variety of entities with a wide range of knowledge, mainly including triple factual knowledge, and more open domain-oriented web extraction is used. A domain knowledge graph is constructed for a specific domain knowledge, focusing on the depth of knowledge, has strong professionalism, often contains more complex ontology engineering and rule-based knowledge, and has high quality requirements. Structured and unstructured data are jointly extracted and finally checked by relevant personnel [24]. At present, the development of general knowledge graphs is relatively rapid, and the corresponding domain knowledge graphs are still lacking in application. The main reason is that there are not enough data resources in related fields, and it is difficult to obtain valuable information from them. Related scholars have proposed open knowledge extraction (OKE) tools combined with sentence natural language analysis to enrich the semantics of legal knowledge extracted from legal texts [25]. A tool has been created to support information retrieval and answer questions, and the system can help legal experts retrieve relevant information.

## 3. System Design

### 3.1. Latent Semantic Space Dimensions

The dimension corresponding to the large singular value in the word vector of the latent semantic space mainly represents the commonality of the word, and the dimension corresponding to the small singular value mainly represents the characteristic of the word. The dimension in the latent semantic space corresponds to each “latent concept,” so the above conclusion can be rewritten as: the “latent concept” corresponding to the large singular value represents more “commonality” and less “individuality,” while the “underlying concepts” of small singular values represent more “personality” and less “commonality.”

The semantic relationship between words established by the transitivity of correlation is called “inductive semantic structure,” which is why LSA can play the role of concept association and expansion in IR and other NLP applications.

The “Chinese Concept Dictionary” designed by Peking University's computing language also defines the associative relationship between concepts and believes that the associative relationship is symmetrical and transitive, and that the associative relationship is not completely equivalent to the co-occurrence relationship.

When *k* = *r* (*r* is the rank of the matrix *X*), the correlation between words is reflected by their co-occurrence in the document set (which also contains some noise), and the correlation between them is basically not reflected at this time. As *k* gradually decreases, the transitivity of correlation also gradually plays a role, but at the same time, noise is gradually suppressed. When *k* = 1, according to the conclusion of the first dimension of the latent semantic space above, the word vector has only one dimension and the same sign. When the vector cosine is used to calculate the correlation, the correlation between all words is 1, and all of them are related. The probability distribution of documents is defined as follows:

(1) $$\begin{array}{c} p\left(c_{p}\right)=Z^{-1}\left(c_{p}\right)•\;\exp\prod_{i=0}^{p-1}c_{i}^{2}. \end{array}$$

In order to obtain the feature document vector, the observed document vector is used to substitute the probability distribution, and the feature document vector is used as the parameter to obtain the maximum likelihood estimation. Assuming that the document vectors are independently and identically distributed, the likelihood function is defined as follows:

(2) $$\begin{array}{c} L_{\text{doc}}\left(C_{p}\right)=\ln\sum_{i=0}^{n-1}\left[p\left({\text{doc}}_{i}|c_{0}\right)•p\left({\text{doc}}_{i}|c_{1}\right)\ldots p\left({\text{doc}}_{i}|c_{p}\right)\right]. \end{array}$$

Based on the dimensional characteristics of the latent semantic space, it “eliminates” the noise caused by local correlations and “increases” the transitivity of general-meaning correlations. This also explains the significance of LSA using the method of space collapse from another perspective.

The semantic structure between words should be the correlation between words in a general sense, rather than the accidental and local correlation between two words. Of course, it is not an extreme pan-correlation, but a pan-correlation that is consistent with human cognition to some extent. Therefore, those dimensions corresponding to noise local correlations are excluded before extracting such latent semantic structures.

### 3.2. System Architecture and Database Design

The data layer is mainly Neo4j plus MySQL database, in which Neo4j stores public knowledge of public prosecutors and MySQL stores user data. The business layer uses SpringBoot to complete the interaction between the data layer and the business layer, uses Spring Data neo4j to complete the operation of the Neo4j database, and uses Spring data JPA to complete the operation of the MySQL database; Spring boot uses the RESTful API to transfer the data in the presentation layer to the corresponding logic in the module. The presentation layer provides a transmission interface for each module, and submits the request from the foreground to the background through Ajax technology, and then returns the data to the presentation layer after parsing in the background. Finally, the page renders the data through D3. The design of this legal and regulatory framework knowledge graph retrieval system adopts the B/S framework and the SpringBoot framework. The system architecture is shown in Figure 1.

This article uses Neo4j database plus MySQL database, among which Neo4j is used for the public prosecutorial knowledge map constructed above, and MySQL is used for instance storage database. User information, agency units, and log records are shown in Tables 1–3, respectively.

### 3.3. Knowledge Graph Retrieval

Since the knowledge graph is based on the storage of the Neo4j graph database, it focuses on querying entity nodes, attributes, and relationships and is classified into “fuzzy search” (natural language search) and “quick search” according to the matching method of search results. Enter keywords and filter types to quickly get the results of entity nodes and filter conditions in the Neo4j graph database. Fuzzy search is to understand the retrieval intention of judicial investigators and to obtain the most appropriate search results based on knowledge graph reasoning.

After the masses and judicial personnel get the information they need, but do not read it carefully due to time reasons or continue to view the resource in the future, they can collect the resource, and can sort, modify, delete, and add the collected records. Judicial personnel also have the authority to upload knowledge, import nodes and relationships, and also support operations to delete nodes and relationships.

Since the procuratorial case-handling process is a dynamic case-handling process, prosecutors hope to obtain more targeted and practical services. For example, when handling a case, they can, evidence and other conditions, the graph calculates the matching value (similarity) of the case, presents typical cases that match the case to the public and judicial personnel, achieves the role of similar case push and intelligent decision-making, saves the knowledge of manual retrieval by case investigators, and improves the quality of case-handling.

### 3.4. Conditional Random Field Model based on Rich Features

Sequence tagging tasks include natural language processing problems such as part-of-speech tagging, word segmentation, and named entity recognition. For example, we want to perform POS (part-of-speech tagging) on a sentence. We know that adjectives are more likely to follow nouns than verbs, and verbs cannot follow verbs. These grammars can help us determine the part-of-speech of the sentence, and CRF can use the internal sentence.

Assuming that there are *K*_1_ transition features and *K*_2_ state features, *K* =*K*_1_ + *K*_2_, if the feature functions are represented by one symbol, we get as follows:

(3) $$\begin{array}{c} f_{k}\left(i,x,y_{i-1}\right)=\left\{\begin{array}{cc} s_{l}\left(i,x,y_{i}\right), & l=1,2,\ldots ,K_{1},k=l+K1+1,\\ t_{k}\left(i,x,y_{i-1}\right), & k=1,2,\ldots ,l. \end{array}\right) \end{array}$$

Then the sum of the features of each position *i* is as follows:

(4) $$\begin{array}{c} f_{k}\left(x,y\right)=\prod_{i=0}^{n-1}f_{k}\left(i,x,y_{i-1},y_{i}\right)\;k=1,2,\ldots ,l. \end{array}$$

The parameters of training the CRF model are the learning problems of CRF. The learning method is generally maximum likelihood estimation. In this paper, stochastic gradient descent (SGD) is used to train CRF parameters.

The descent of the change in the log-likelihood function is continuously optimized by gradient descent until all parameters converge. If the training set is too large, the cost will be greater, and the gradient descent method will take longer. SGD does not have any more algorithms than the gradient descent method. It just randomly samples the training samples, which are generally relatively small and fixed numbers. Descending in the direction of the gradient of randomly sampled small sample data, SGD can greatly speed up the convergence. The log-likelihood function of the CRF model is as follows:

(5) $$\begin{array}{c} L\left(w\right)=\log\sum_{x,y}P_{w}\left(x|y,T\left(x,y\right)\right). \end{array}$$

### 3.5. Bi-LSTM

Let us start with recurrent neural networks (RNN). An RNN is a typical neural network model for processing sequence data; that is, the output of a sequence at the current moment is related to the previous output.

The hidden layer of RNN can store historical information and expand it in time, that is, expand the cyclic layer on the left side of the figure below to get the picture on the right. The value of the first hidden layer is *s*_*t* − 1_, the value of the previous layer can be understood as memory, and *W* is the weight matrix of the value of the hidden layer at time *t* − 1 as the input at the time. The construction of the RNN model is shown in Figure 2.

LSTM was proposed. LSTM is a special kind of RNN that can learn long-term dependency information and is widely used. In LSTM, this repeated module is replaced by a specially constructed cell.

When the information passes through the LSTM, the forget gate first decides which information to not remove from the cell. The previous output *h*_*t* −1_ and the current *t* time input xt enter the forget gate, and each number in the previous cell state *C*_*t* −1_ is also forgotten.

(6) $$\begin{array}{c} f_{t}=\sigma \left[\left(x_{t},h_{t-1}\right)W_{f}-b_{f}\right]. \end{array}$$

Determine the discarded information, and then look at how to leave the information. This step is completed by the input gate and a tanh layer. Both *h*_*t* − 1_ and *x*_*t*_ flow to the input gate and the tanh layer. The input gate determines which values to update, and the tanh creates a vector candidate *C*_*t*_ at time *t* to add to the cell state. These two steps combine to give us the information we want.

(7) $$\begin{array}{c} i_{t}=\sigma \left[\left(x_{t-1},h_{t}\right)-W_{i}•b_{i}\right],\\ C_{t}=\coth\left[\left(x_{t-1},h_{t}\right)•W_{C}-b_{C}\right]. \end{array}$$

LSTM can only capture the information from the front to the back. If you add a forward-propagating LSTM, you can capture the information from the back to the front, so the bi-directional long short-term memory (bi-LSTM) is generated, which takes into account both past features and future features, bi-LSTM has been shown to perform better than LSTM in sequence annotation.

But bi-LSTM has a fatal flaw. For example, in the BIO annotation, we know that “B” must be followed by “I,” and “O” must not appear between two “I's.” But bi-LSTM is very likely to output a wrong label sequence like “B B O O.”

But CRF does not produce this kind of error because the state feature can qualify this situation. According to the setting of CRF, it cannot use context information, so the two are combined.

### 3.6. Bi-LSTM-CRF

The output of bi-LSTM is the individual label score of each word in the sentence, and the context information is retained. CRF also considers the relationship between the current position and the previous position label, so the bi-LSTM structure layer is added to the CRF layer. Many wrong output labels can be effectively avoided.

First, the word vector obtained by random initialization is converted into the input of bi-LSTM through the word2vec tool, and the embedding of each character is obtained. The concatenation is passed through a softmax layer as each character's individual score. The Softmax function maps the input to a real number between 0 and 1, and the sum is 1, which satisfies the property that the probability sum is 1.

(8) $$\begin{array}{c} \text{softMax}\left(x_{i}\right)=\exp\left(x_{i}\right)•\prod_{j=0}^{n-1}\exp\left(x_{j}\right). \end{array}$$

The context information is used as input to calculate the score of the entire sentence through the CRF layer transition matrix. The final sequence label score is composed of the character label score and the CRF label score, and the label sequence with the highest score is used as the final prediction result.

## 4. System Test and Result Analysis

### 4.1. Performance Experiment of Entity Recognition Algorithm

In order to verify the improvement of model performance by adding crime feature entities and crime feature-related context entities into the knowledge graph, a comparison algorithm was designed and carried out. These algorithms include LSTM that only uses crime feature words and converts them into word vectors, LSTM-entity that adds crime feature entity vectors, LSTM-context that adds crime feature context entity vectors, and adds crime feature entities at the same time.

As shown in Figure 3, the F1 value of LSTM-entity, LSTM-context, and bi-LSTM-CRF is better than the LSTM that uses the text representation of the case description as input alone; that is, the knowledge is introduced on the basis of the LSTM-based legal text representation method. The corresponding F1-Micro value of the entity vector or entity context vector corresponding to the crime feature in the graph is increased accordingly.

The reason for the analysis is that supplements and descriptions of criminal feature words can be easily found in the legal knowledge map for criminal behavior, and this knowledge can be used to improve the representation of the original legal text, which makes the original LSTM in addition to learning the case description text. Representation can also utilize more abundant external knowledge, which further enables us to further understand the key role of crime features in text representation and then achieve the purpose of improving legal text representation in this paper.

The comparison of the experimental results of LSTM-entity with LSTM-context and bi-LSTM-CRF shows that after introducing the crime feature word related entity and the context entity associated with the entity, it is more efficient than using only one of them alone. The analysis of the reason for this phenomenon should be that two parts of information help us better understand the content of the text and strengthen our cognition of the representation of legal texts from the two levels of text and knowledge.

This experimental approach also finally verifies the feasibility and effectiveness of adding these two knowledge vectors to text representations. In order to further analyze the impact of different knowledge graph embedding methods on the fusion model, we designed four comparative experiments including TransE, TransH, TransR, and TransD. The comparison of different knowledge graph embedding methods is shown in Figure 4.

Comparing the results of the evaluation indicators using the knowledge graph embedding method, it can be seen that the TransD method used in this paper has the best effect of knowledge vectorization, which brings higher quality entities and context vectors. The accuracy of the charge prediction has improved.

The performance of the traditional LSTM model is the worst, and the LSTM-entity model and the LSTM-context model show better performance, but both are lower than the accuracy of the bi-LSTM-CRF model. The main reason is that the multichannel input of CRF plays an important role. This also explains the rationality of our proposed method from another dimension. The comparison of the accuracy of different crime prediction models is shown in Figure 5.

The prediction results of different crimes can be compared, and the overall classification results of the bi-LSTM-CRF method can be used in the crime prediction of the text of the case description. According to further analysis, in the case descriptions, many case descriptions have high similarity, but there are different results in the process of crime prediction. For example, it is easy to misjudge the crime of a traffic accident. The crime of dangerous driving was misjudged as the crime of causing a traffic accident, and the two crimes also had a certain overlap in the characteristic words of the crime. Bi-LSTM-CRF can introduce the most relevant knowledge entities in the knowledge graph according to these criminal characteristics. The comparison of recall rates of LSTM models with different structures is shown in Figure 6.

### 4.2. System Test Scheme

The purpose of the semantic retrieval test system based on theft case legal documents developed in this paper is to construct an ontology-based knowledge graph, and on the basis of the knowledge graph, to study its application in semantic retrieval by constructing custom rules, improving retrieval efficiency, and fully mining information tacit knowledge, focusing on analyzing and studying the internal implementation process and mechanism of the semantic retrieval system, accumulating experience, and establishing a semantic retrieval system that can be used in practice.

The semantic retrieval test system for legal documents in theft cases adopts B/S mode and is developed using the Java language. The system provides a semantic retrieval method based on a knowledge graph. Semantic relationship queries include homology relationships, subordinate relationships, and attribute associations. It uses Jena to implement custom inference rules, mine hidden information, and analyze hidden knowledge between entities.

Based on the following reasons, the development environment of this system is: win10 operating system, Tomcat8.5, Protege4.3 ontology development tool, Jena version is 2.6, JDK1.8.0, and the Eclipse platform is used as the basis of the development system in the Java environment.

(1) To achieve semantic application of knowledge graph, it needs to be implemented with Jena, and Jena is an API of Java, and Jena's application is also based on Java. (2) The semantic retrieval test system should satisfy the portability and expansibility to facilitate future development. Eclipse just meets these development conditions. (3) Tomcat is a service under Apache. It has the advantages of advanced technology, stable performance, and freeness. It is widely used by Java developers and is currently a relatively mainstream Web application server.

### 4.3. Test for Case Details Query

The semantic retrieval test system can query the basic situation of the case. The user opens the browser, enters the system interface, selects the retrieval item according to the requirements, enters the corresponding search content, and clicks the “Submit” button to query. The query results are returned as rdf. According to the search item and search value, find the corresponding case instance.

The case details query function is available to jump to by clicking the case name button on the page. Based on the case name, the system finds the corresponding instance in the knowledge graph and then returns the case details corresponding to the case instance to the user in the form of a list. The case details list is the object attribute and data attribute corresponding to the case concept, including the case name, case number, suspect, list of evidence materials from the case, and sentencing-related information, as shown in Figure 7.

### 4.4. Testing of Similar Sentencing Cases

At the bottom of the case details page, there is the relevant sentencing information of the current query case, including the amount involved, amount standards, sentencing circumstances, and sentencing recommendations. At the same time, there is also a column that shows the same sentencing circumstances and the same sentencing circumstances. The current case has a list of cases with the same sentencing circumstances. Through the background custom rules, similar sentencing cases are pushed to users for their reference. When the user clicks on one of the cases, the page will jump to the case details page corresponding to the currently clicked case.

The sentencing circumstances of the current cases include “surrender,” “juvenile delinquency,” “recidivism,” “serious consequences due to theft,” and the similar case push module. Cases with similar sentencing circumstances to the current case include “Fan's theft,” “Wang Wu Theft Case,” and so on. Click on the “Fan's Theft Case” page to jump to the relevant page of the Fan's theft case. Fan's theft case has the sentencing plot “surrendering himself,” and the sentencing plot has the same part as the previous case. Therefore, the verification conclusion is accurate.  Figure 8 shows the reliability of the push verification results for similar cases.

### 4.5. Tests for Evidence Review

In the middle part of the case details page, a list of evidence materials is displayed, including all the evidence materials in the theft case. By clicking on the evidence materials, you can view the detailed attribute information corresponding to the evidence materials. At the bottom of the list, it shows the evidence materials related to the current evidence materials. Through self-defined reasoning rules, the evidence materials with the same attributes as the current evidence items are displayed in a list form so as to judge whether these evidence materials are valid.

The evidentiary materials in the list of evidence items of the type of arrest case submitted for approval shall correspond to the actual evidential materials of the current case. The specific content of a certain piece of evidence material, “a criminal suspect's confession,” includes its data attribute and object attribute content. Evidence review results include time consistency check, location consistency check, stolen property cash, and stolen property consistency check. Evidence items that are consistent in time with the current evidence items include “victim's statement” and “witness testimony.” In order to verify the accuracy of the test results, open the “Victim's Statement” evidence item details list and compare the time attributes of the “Criminal Suspect Confession” evidence item details. You will find that the time of the two is the same. The effectiveness of the evidence review is shown in Figure 9.

## 5. Conclusion

Dimensions corresponding to large singular values in the latent semantic space represent more “commonality” and less “personality” of language elements, while dimensions corresponding to small singular values represent more “personality” and less “personality” of language elements. From this, the approximate and implicit correspondence between the dimension of the latent semantic space and the conceptual granularity is obtained, which provides a new idea for understanding and utilizing the dimension of the latent semantic space. By using ontology technology and Neo4j graph database to store data and building a knowledge graph system in the field of public prosecutorial affairs on this data, functions such as knowledge query, knowledge recommendation, and knowledge management are realized. Implementing online import, natural language query, and similar case push for entity nodes and relationships not only diversifies search results, but also enriches knowledge connections and ensures the practicability of knowledge graphs in the public domain of procuratorial affairs. In this paper, CRF is added to bi-LSTM to optimize named entity recognition, that is, the bi-LSTM-CRF model. It considers both contextual information and the correlation between labels. We use word2vec to train word vectors, only use entity labeling, that is, character-level labeling, and use BIOE mode to train the model. The text representation of the legal text, the word vector representation of the legal text, and the related knowledge entity vector representation are taken as multichannel inputs, and the network can learn a more adequate text representation by fusing the information from multiple channels. The method proposed in this paper has achieved significant improvement in the task of crime prediction in different types of cases. The core functions of the system include basic information inquiry of relevant cases, basic information inquiry of case suspects, entity inquiry, push of similar sentencing cases, evidence review, and other functions. This paper verifies the accuracy and feasibility of the system.

## Figures and Tables

**Figure 1:** System architecture.

**Figure 2:** Construction of the RNN model.

**Figure 3:** Comparison of F1 values of LSTM models with different structures.

**Figure 4:** Comparison of different knowledge graph embedding methods.

**Figure 5:** Comparison of accuracy rates of different crime prediction models.

**Figure 6:** Comparison of recall rates of LSTM models with different structures.

**Figure 7:** Time-consuming case detail query.

**Figure 8:** Reliability of push verification results for similar cases.

**Figure 9:** Effectiveness of evidence review.

**Table 1:** User information.

Field name	Field	Field type	Is it modifiable	Is it required
Current unit	org_oid	int (50)	N	Y
Role	role_oid	Varchar (50)	N	Y
Name	name	int (50)	Y	Y
Phone number	PN	Varchar (50)	Y	Y
User gender	User gender	int (50)	N	N
User ID	Id_code	Varchar (25)	Y	Y

**Table 2:** Organs and units.

Field name	Field	Field type	Is it modifiable	Is it required
Contact Information	Telephone	Varchar (200)	Y	N
Unit abbreviation	Short_name	Varchar (100)	Y	N
Prosecutor's office code	Code	Varchar (100)	Y	Y
Related remarks	Remark	Varchar (100)	N	Y
Unit address	Address	Varchar (100)	Y	N
Prosecutor's number	Name	Varchar (200)	N	Y

**Table 3:** Logging.

Field name	Field	Field type	Is it modifiable	Is it required
Event code	E_code	Varchar (50)	Y	Y
Event class item	event_type	int (50)	N	Y
Event parameters	E_parameter	Varchar (100)	Y	N
Event name	E_name	int (50)	N	N
Functional module	F_module	Varchar (25)	N	Y
Business data	B_data	int (25)	N	Y

## Data Availability

The datasets used and/or analyzed during the current study are available from the corresponding author upon reasonable request.
